This article has been retracted.

# The Application of Color Psychology in Community Health Environment Design

**DOI:** 10.1155/2022/7259595

**Published:** 2022-08-25

**Authors:** Jicheng Yang, Xiaoying Shen

**Affiliations:** ^1^School of Design, Beijing Normal University, Zhuhai, Guangdong 519087, China; ^2^Wuxi Vocational College of Science and Technology, No. 8 Xinxi Road, Wuxi, Jiangsu 214000, China

## Abstract

The topic of health has gained importance in today's society in the context of a healthy China. The success of community environmental design is intimately correlated with everyone's physical and mental health since it is the setting for people's daily lives. At present, although the facilities and equipment of the community environment in our country are improving day by day, the important role of color psychology in the community environment has been neglected. Color has always been a part of human life and a very important component of the community environment. When it comes to the design of communal environments, the color design of various areas will have variable degrees of influence on the psychological space and perspective of individuals. Therefore, the purpose of this paper is to investigate the application value of color psychology in the design of community health environments using color psychology as a scientific foundation. Additionally, the paper attempts to use color psychology as a scientific basis to study the thinking of health issues in the community environment. In addition, the results of the questionnaire survey are used to perform analysis and discussion in order to investigate the regular characteristics of the various research objects, as well as their preferences and psychological needs for color. This is done with the goal of providing empirical support for the improvement of the community environment and the health of the people living in it. In the end, the results of the questionnaire survey are compiled with four different design concepts. These design principles include functionality, naturalness, beauty, and safety. And the design intention and optimization strategy from the three directions the overall building, planting, and paving in the community healthy environment are then presented. This is done in order to create a colorful and comfortable healthy environment for the community life of people and to support the development of people's physical and mental health.

## 1. Introduction

The growth of modern industrial cities has contributed to deterioration in the quality of the living environment in which people live, which in turn has led to a number of issues relating to public health. Residents of metropolitan communities are increasingly concentrating their attention on health concerns. The biopsychosocial medical concept suggests that the environment (both physical and social) in which an individual lives has a significant impact on both the individual's mental and physical health. Community, as the most fundamental component of urban planning, serves as an essential space carrier for the daily activities and social interactions of its members. It is not just one of the factors that contribute to issues with mental health, but it is also an essential venue for the improvement of the inhabitants' mental health [1]. According to the community environment and health relationship model proposed in literature [2], the individual characteristics of inhabitants are thought to be the primary determinants of their mental health. Both the community's social and physical environments can have an effect on the people' mental health. This is especially true of the former. To put it another way, in order to protect people's health, we need a healthy environment. It is self-evident how important the environment of the community is to the health of its residents, and it can have an effect on the health of the entire city as well as its residents.

In addition, as a result of the growth and advancement of society as a whole as well as the increase of community residents' health awareness, the aspiration and yearning of community residents for a healthy community have become increasingly acute. Therefore, in the context of a healthy China and healthy cities, the question of how to break through the current community construction, which primarily focuses on the renewal of physical spaces such as buildings, has become an urgent problem that needs to be solved. At the same time, thinking about community environmental design issues from the perspective of health and from a deeper and more comprehensive perspective is essential. At the moment, it is turning into a hot point for study in order to improve the community environment, exert community health efficiency, improve public health status, and promote well-being for the members of the community by means of environmental intervention. The planning and design of green open space will bring direct health advantages to urban residents, according to research [3, 4], and studies have demonstrated that people's health is affected by the design of natural environments [3, 4]. In addition, a number of studies have demonstrated that having access to green space in a community can improve people's physical, mental, and social health [5].

Therefore, to design a healthy community environment, it is necessary to deal with the relationship between people's psychology, physiology, and various spaces. Color is a very important component of the community environment. The study of color on people's psychology and behavior can help improve people's activity experience in different environments [6]. In the early days of human development, human beings realized the special charm of color, and at that time they began to use color to decorate life. The discovery of the seven-color spectrum gave humans a deeper understanding of color, and people gradually realized the influence of color on people's psychology, and color psychology was born [7]. Color psychology is a science that studies the relationship between color and people's psychology. In recent years, more and more research has been carried out in the field of color psychology, and it has been widely used in many fields, further deepening people's understanding of lifestyle and life values [8, 9]. Literature [10] expounds the relationship between color and space from the three perspectives color, greening, and furnishings and applies relevant theories to practical projects. They hope to use color, green vegetation, and space to design a plan for an office leisure area with a “healing system” effect. Literature [11] discusses how to combine it with urban road greening design by analyzing the relevant theoretical knowledge of color psychology. According to the psychological characteristics of users and the psychological effect of color, a humanized urban road green space is designed. Literature [12] studies the application of color psychology in hospital interior design. From the perspective of color psychology, the author conducts sufficient research on color and psychology of indoor design and analyzes how to use color psychology in hospital indoor design. Literature [13] carried out space color design from the perspective of old-age care, focusing on analyzing the particularity of old-age buildings. They make full use of the theoretical basis of color psychology and color physiology and analyze various design problems of old-age buildings and indoor public spaces from the perspective of color design and then hope to use the role of color to effectively affect the psychology of the elderly.

To sum up, color is the main factor affecting the human senses and also affects the physiology and psychology of the human body. It will inevitably affect the effect and function of the community environment design. Therefore, in the design of community health environment, it is necessary to deeply study the principles of color psychology in order to better meet people's psychological needs. But at present, it still lacks scientific theoretical guidance for the color design in the community environment of our country. The existing research on the color design of the community environment is still immature, and there are differences in the application of color in the community environment, and a complete color system has not yet been formed. In view of this, through the research of related theories, this paper tries to design the community health environment based on color psychology. Through the effective combination of the two, the principles and strategies of community health environment design under the guidance of color psychology theory are proposed. The main research contents of this paper are as follows: first, the application value of color psychology in community health environment design is discussed; second, through the method of questionnaire survey, the regular characteristics of different research objects, their preferences and psychological needs for color are explored, so as to provide empirical reference for community environment optimization and population health; and finally, combined with the results of the questionnaire survey, the design principles and optimization strategies of community health environment under the guidance of color psychology are summarized. It is hoped that through the research of this topic, the color design in the community health environment will be enriched, and a healthy, natural, and comfortable community color space will be created, in order to create a high-quality, high-level living and leisure and entertainment environment for people, promote people's physical and mental development, and ultimately realize the beautiful vision of a healthy China.

## 2. Related Theory

### 2.1. The Concept and Development of Color Psychology

A significant subfield of psychology and a rising academic field, color psychology is becoming increasingly popular. The primary focus of color psychology is the investigation of the impact that color has on the psyche and behavior of humans [14]. Color is capable of fully expressing a wide range of human emotions, and the combination of brightness and color is the source of all visible phenomena. Through human visual contact, color will have many different and complicated effects on people's psychology, physiology, and imagination. Additionally, people's psychological and physiological states will affect how they perceive and think about color. According to the theory of color psychology, different hues are thought to have varied effects on the psychology and emotions of people, and certain regular causal correlations are considered to exist between colors and the psychological reactions of people. In addition, in terms of its emergence and progression, color psychology has gone through a period of rapid expansion, which has been primarily driven by the advancement of economic growth. The Munsell color system in the United States [15], the Ostwald color system in Germany [16], and the PCCS (practical color coordinate system) color system in Japan [17] are the most extensively diffused and used systems in the world as far as is known about color psychology's extant theoretical systems.

Although the current research on color psychology is still immature, it has not been formally defined in the research of psychology. It is undeniable that its influence on human psychology exists objectively and is spontaneously applied to real life by human beings. For example, shopping malls use color matching to upgrade their brand, attract customers, and increase their desire to buy. The restaurant and bar use color matching to create their atmosphere and highlight the characteristics. In addition, color psychology has also been widely used in architectural design, painting, graphic design, animation, industrial design, etc. [18–20]. There is also color therapy in medicine, that is, using the psychological effects of color to carry out adjuvant treatment at different levels for patients [21].

### 2.2. The Main Theories of Color Psychology

#### 2.2.1. Color Emotion

Colors are able to communicate not just visual information but also feelings. One of the functions of color is to convey a range of feelings to people while also providing them with a striking visual impression. The field of color psychology has conducted pertinent study on the laws of people's psychological effects on color. This research has provided a scientific basis for us to assess and create colors in community health environments, thanks to the work that was done in color psychology. The human imagination and memory can be stimulated by color, which can then further raise human emotional resonance.  Figure 1 provides a synopsis of the psychological qualities associated with a selection of representative colors.

#### 2.2.2. Symbols of Colors

The sign of color is the reflection of the mental spectrum of color that is contained in a single hue. It is a reference to the unique connotation that is exhibited between a hue that is widely recognized and the items that are linked with it. On the other hand, people from different eras and walks of life have a tendency to ascribe diverse symbolic meanings to certain hues. It is possible to say that the symbolism of color not only originates from humanism with historical and cultural legacy but also exists in society as a symbolic form. This is something that can be said since it is something that can be said.  Table 1 provides a common metaphorical interpretation for each color.

#### 2.2.3. Character Traits of Color

Each color is a complete individual. If anthropomorphic, they represent different characters and have their own personalities. Referring to the relevant color psychology theory, this paper summarizes the personality characteristics represented by each color, as shown in Figure 2.

## 3. Investigation and Analysis of Community Health Environment Design Based on Color Psychology

### 3.1. Research Objects and Methods

#### 3.1.1. Research Object

During the period from March 2022 to June 2022, with the mobilization and assistance of local community staff, the random sampling method was used to recruit local community residents from 10 communities in City A as research object. Paper questionnaires were distributed to them, of which 5 communities or streets were selected in urban and suburban areas. The definition of local residents in the study is as follows: they have the household registration of the local permanent population, have lived in the community or street for 1 year or more, and are between 18 and 75 years old. After a detailed explanation of the purpose of this research study, participants completed a self-administered questionnaire anonymously on the basis of written informed consent. If they have difficulty filling it out, it would be guided by trained investigators.

#### 3.1.2. Questionnaire Design and Survey

A set of questionnaires was designed in the study. The survey content involves the age, occupation, gender, and other basic information of the respondents, as well as their preference for color, the impact of different colors on their emotions, and their inclination to the color of the ideal community space. Through the research, three characteristics of the regular characteristics of different respondents, their preference for color, and their psychological needs for color are summarized.

#### 3.1.3. Quality Control

After the research subjects completed the questionnaires, the trained project team members were responsible for the quality control of the questionnaires. The questionnaires with unreasonable logic, too much missing information, and too many consistent responses were eliminated. In the end, a total of 100 questionnaires were distributed and 89 valid questionnaires were collected.

### 3.2. Result Analysis

#### 3.2.1. The Regular Characteristics of the Research Object

*(1) Basic Situation.* A total of 100 questionnaires were distributed in this survey, and 89 valid questionnaires were collected. Among the valid questionnaires, there were 38 males and 51 females, accounting for 42.7% and 57.3% of the total, respectively, as shown in Figure 3. Due to the random distribution of the questionnaires, the ratio of males to females was not controlled artificially. In addition, the mean age of the research objects was (45.29 ± 15.35) years old.

*(2) Education and Career*. In terms of educational background, the percentage of high school and technical secondary school (57.3%) is the highest, and the proportion of junior high school and below is 9%, and the proportion of university and above is 33.7%, as shown in Figure 4(a). Since the vast majority of the research subjects have not received higher education, their cognition of color is still at the level of whether they look good or not. Combining the occupational proportions in Figure 4(b), according to the survey report, among the survey respondents, government departments, service industries, and manufacturing industries have the highest proportions.

#### 3.2.2. Research Objects' Preferences for Color

In the questionnaire designed in this paper, there are two questions: “What is your preferred color?” and “What is your preferred color tone?” The purpose is to explore the preferences of the research objects on the hue, lightness, and purity of colors. Data statistics were carried out for the selection of different age groups, and the statistical results of the hue, lightness, and purity of the colors of different survey groups were obtained, as shown in Figure 5 and Figure 6, respectively.

As shown in Figure 5, according to statistics, in the hue selection, the number of yellow selections is the most, with a total of 65 times. Hue selection frequency in descending order is as follows: yellow > green > red > blue > orange > purple > white > black. Moreover, respondents of different age groups have different preferences for hue. Young people are more inclined towards green, blue, black, and white. Middle-aged people prefer green, blue, and yellow. The elderly prefer brighter colors such as red, orange, yellow, and green and do not like dark or dark colors such as black and white.

As shown in Figure 6(a), among the lightness selections, the number of medium lightness selections is the largest, 45 times in total. The lightness selection frequency in descending order is as follows: medium lightness > high lightness > low lightness. Similarly, as shown in Figure 6(b), among the color purity selections, the medium purity selection is the most frequent, with a total of 49 times. The purity selection frequency is sorted from large to small: medium purity > high purity > low purity.

#### 3.2.3. Research Objects' Psychological Needs for Color

*(1) Character Analysis*. According to the survey analysis, most people tend to be low-key and restrained, as shown in Figure 7. Therefore, in the design of community health environment, in order to relieve people's tension, anxiety, and depression, more warm, bright, and soothing colors should be used to provide people with a comfortable and relaxing activity environment.

*(2) Sentiment Analysis*. According to the analysis of the survey questionnaire, the categories that account for the biggest proportion of respondents when people feel anxious, lonely, and emotionally unstable are presented in Figure 8 as having the orange-yellow, blue-green, and red-pink color combinations. This demonstrates that various respondents have a tendency to favor warm colors when they are not in a good emotional state. The color combinations black-white and blue-purple were the ones that received the fewest votes, with only 4% and 3% of the total, respectively. This demonstrates that people are most likely to feel dejected and melancholy when exposed to any of these two hues. As a result of this, it is clear that the indoor humanistic space of the community healthy environment should select colors that are vibrant, bright, and cheerful. Green is the color that should be used for the natural outside surroundings. These hues have a calming effect on people by easing their anxious feelings. In addition, it should not use dark, intense hues like dark purple, dark coffee, dark green, dark blue, or dark gray. These colors should be avoided.

*(3) Image Analysis*. As shown in Figure 9, according to the analysis results, most of the survey respondents tend to choose a warm, soft, relaxed, safe, and happy ideal community environment, and fewer people choose a serious, rational, and stable environment. As the current pace of life is getting faster and faster, people's pressure has become greater and greater. They prefer a comfortable and natural environment and pursue the concept of tranquility, far-reaching, and natural behavior. Therefore, the color design in the community health environment should also be warm, soft, soothing, and bright.

Based on the above analysis results, the design style of the interior space in the community environment can be chosen to be more natural. Log-colored wood and milky white latex paint can be used for large-area decoration, and then personalized design can be carried out in different areas according to the color preferences, emotions, and imagination of different groups of people, so as to meet the activity needs of different groups of people.

## 4. Community Health Environment Design Strategy Based on Color Psychology

When combined with the findings of the analyses of the previous questionnaires, as well as the theory of color psychology and the premise of adhering to the principles of aesthetics, safety, naturalness, and functionality, the design intention and optimization strategy are proposed in three aspects from the building, planting, and paving in the healthy environment of the community. These three aspects include building, planting, and paving. It is anticipated that the colors that are used in the community environment of our country will become more harmonious, comfortable, and beautiful. This will result in the creation of a community environment that is helpful to the leisure and amusement of the people.

### 4.1. Design Principles

#### 4.1.1. Aesthetic Principles

When it comes to the planning of healthy settings for communities, color plays an important role. It is both an artistic expression and a manifestation of the human spirit in the context of the community in which it takes place. People can have a more calm and enjoyable time participating in activities if the colors and aesthetic design elements are coordinated well. The following is a list of aesthetic criteria that should be considered when designing color schemes for community health environments: (1) constancy amidst dynamic motion. The term “unity” most often refers to the uniformity of the primary color that is shared by the color of the building facade and the color of the pavement. The shift focuses mostly on the tonal alterations that are supplemented by the color of the gaming facilities and the color of the plant landscape. To put it another way, the color design of the community health environment is one in which unity and change coexist and accommodate themselves to one another; (2) a combination of contrast and harmony. The concepts of unity and change can be best embodied by contrast and harmony. The contrast of colors has the potential to enhance the impression of contrast that exists between the colors of the various parts of the communal environment. The harmony of colors has the potential to make the colors of the various aspects of the environment appear more similar and harmonious, and it also has the potential to improve the overall impression of the color of the community's environment; and (3) a sense of symmetry and equilibrium. One of the distinguishing features of Chinese art is its emphasis on symmetry and balance. Since ancient times, this aesthetic theory has been the one that has been employed in design projects the majority of the time. People's bodies and minds can be adjusted through the use of the principle of symmetry and balance in color design in community health environments, which also helps create an atmosphere that is cozier, more relaxing, and filled with opportunities for action.

#### 4.1.2. Security Principles

At present, the proportion of people suffering from depression, anxiety, youth myopia, obesity, and other psychological and physical diseases is increasing year by year, affecting people's physical and mental health. Creating a safe and healthy community environment is increasingly important. Although with the improvement of various facilities and equipment in the community environment in our country, it has high safety. However, there is a lack of research guidance and normative requirements for the safety of colors. Therefore, safety design principles should also be an important consideration in designing community health environments. The primary purpose of the safety principle of color design is to pay attention to the color synesthesia effect of community environment color on people and to create a healthier and more comfortable community environment. First of all, it is necessary to rationally apply color and its basic attributes to avoid color pollution in the community environment. Second, the safety of community indoor activity space should be fully considered. For example, in material selection, nonirritating, nonpolluting environmentally friendly materials are used. On the ground pavement, the complementary or contrasting relationship of colors is used to satisfy the spatial orientation. In the guidance and identification, the color system is used for safe instruction guidance and evacuation.

#### 4.1.3. Naturalness Principles

In the color design of community health environment, special attention should be paid to the principle of naturalness of color design. The beauty of many natural landscapes cannot be described in words but can only be experienced personally. By designing large areas of lawns, sloping land, flowers and trees, etc., the number and area ratios of natural landscape colors in community landscape colors are increased, so that people can fully contact nature, so as to cultivate people's sentiments and relax their mood. Studies have shown that, compared with artificial colors commonly used in buildings and pavements, plant landscape colors are more diverse and have seasonal changes. Therefore, the natural principle of community healthy environment design is to change the original design mode, enrich the natural plant landscape in the community, and strengthen greening. In addition, the color elements of different landscapes in the community environment should be matched with each other, while increasing the application of natural colors in building facades, paving, and game facilities.

#### 4.1.4. Functional Principles

Community health environment not only includes outdoor sports and fitness, children's games, and other places but also has many other functions, such as indoor games and entertainment, gathering and distributing activities, sports, and reading and learning. Different functional areas have different requirements for color design. At the same time, color can affect the warmth, light and shade, and volume of a space. Therefore, in the design of community health environment, it is necessary to adhere to the functional principle, make full use of the characteristics of color to serve the space function, and make the color and the space where it is in harmony and unity.

### 4.2. Specific Strategies

#### 4.2.1. Optimal Design of Overall Architectural Color

The architectural color design of community activity venues is the guidance and representative of the overall culture and style of the community and is the main form of displaying community creative design. At present, the architectural color design styles of common community activity venues in China include colorful, simple, and blank. The choice of building color in the community can be summarized into three parts: background color, theme color, and key color. The background color generally chooses a uniform tone, with a soft combination of hue, saturation, and lightness, which is mainly used in the ceiling, floor, wall, and other large space finishes. The theme color is the main color of each functional area, and different areas should choose different hues based on the visual and psychological states of different groups of people. The key color has the role of embellishment and emphasis in the collocation. Most of them use color combinations with very large contrast and strong contrast. It is generally used in forms that require people to pay special attention to identification, and it plays the role of finishing touch in the space.

#### 4.2.2. Optimal Design of Plant Material Color

The colors in nature are the most abundant, and the design of the plant landscape should conform to the principle of color complementarity. Plants exist in nature. They not only purify the air and adjust humidity but also beautify the environment where they are located. In addition, plants can interact with people, while green and yellow plants are beneficial to people's eye health and relieve visual fatigue. Therefore, appropriately increasing the green area in the community environment can make the indoor and outdoor look more dynamic. It can also reduce people's sense of loneliness and loss and bring people closer to nature. Different colors of plants can also cause different feelings. For example, green itself has a calming effect, so many hospitals also use green plants as the embellishment of the environment. Red flowers can make people feel more enthusiastic, while white flowers make people feel elegant. Yellow flowers can make old people feel good. Therefore, the ecological and interesting nature of the community environment can be enhanced by creating a unique natural landscape.

#### 4.2.3. Optimal Design of Paving Color

When people play games, the first environmental information received in the brain is the color of the pavement. Therefore, the pavement color design in the community environment is very important. It can be said that the design of pavement color is the key to the overall color of the community environment. It has the integration of various landscape elements. The design of pavement color can increase the activity of the space through the color tone and transition the overall color matching of the landscape, so as to connect different spaces in the community environment. For example, when selecting the sign material for the community indoor environment, through the unique sign material and the reasonable matching of colors, the softness and cleanliness of the space can be fully displayed.

As mentioned above, the color optimization design of each component in the community environment should ultimately form the consistency of color application. By combining the principles of color psychology and the color design principles of community health environment, and integrating the overall architecture, plant materials, and pavement elements in the community environment, a color optimization strategy for the community health environment is proposed to improve the monotony and proportion incongruity of colors in the current community environment. Through the selection and matching of colors, the activity space is more clearly defined, the environment of the community is improved, and a new type of community health environment with high appearance, high level, and comprehensive benefits is created.

## 5. Conclusion

A community environment that meets health demands is an essential demand of modern community development in the context of healthy China, and it is also an unavoidable trend of future community development. Color is inextricably linked to people's daily lives. Color can be reflected as a language in the human neurological system, activating and influencing people's thoughts and feelings. Color, in other words, is directly linked to people's psychological feelings. As a result, when color is used in community environment design, the color design of different activity spaces will have distinct effects on people's psychology, physiology, and mood. Simultaneously, as color psychology research advances, we become more conscious of the critical function that color plays in people's daily lives. As a result, the focus of this research is on how to combine color psychology with community health environment design to better meet the physical and mental health needs of different groups of color, in order to create a color-comfortable and warm community environment and improve residents' health. This study begins with color psychology, then integrates people's life and spiritual demands, and then successfully blends color psychology with community health environment design to produce a more comfortable and acceptable community activity space. The community environment may not only meet people's everyday requirements, but also their spiritual wants, as well as holistically improve their bodily and mental health.

Although this research has achieved phased results, there are still some problems that need to be further improved and optimized. First, at the theoretical level, this paper simply analyzes the role of color psychology in community health environments. However, there are many elements involved in the construction of a healthy community environment. In the future, we can learn from domestic and foreign research experience and consider factors such as walkable space, natural environment, public service facilities, and the needs of special groups as important content of the construction of a healthy community environment. Second, at the research level, the questionnaire survey employs the random sampling method to recruit research subjects in the community. Moreover, the recruited research subjects ignored the special needs of children and adolescents, and the sample representation was insufficient. In view of this, the follow-up research can consider designing more complex scales, introducing indicators such as health variables, and conducting more in-depth research on different populations and different types of communities. Therefore, combined with more targeted research conclusions, it provides more accurate strategies for the design and optimization of community health environment and constantly enriches and improves the practice cases and basic theories of healthy community building under the “Healthy China” strategy.

## Figures and Tables

**Figure 1:** Emotional characteristics of several representative colors.

**Figure 2:** Character traits of color.

**Figure 3:** Male-to-female ratio among respondents.

**Figure 4:** Statistics of educational background and occupation of the respondents. (a) The percentage of educational backgrounds among survey respondents. (b) The percentage of different occupations among survey respondents.

**Figure 5:** Statistics on hue preference of different respondents.

**Figure 6:** The choice of brightness and purity for different respondents. (a) The choice of brightness of different respondents. (b) The choice of purity of different respondents.

**Figure 7:** Character statistics of respondents.

**Figure 8:** Color preferences of respondents when they are emotionally unstable.

**Figure 9:** The ideal living environment image of the respondents.

**Table 1:** The common symbolic meanings of some colors.

Color	Symbolic meaning
Red	Festive, excited, passionate, dangerous, loving, auspicious, gaudy, enthusiastic, awe-inspiring
Dark red	Noble, solemn, selfless
Pink	Gentle, soft, earthy, reserved
Lavender	Elegant, romantic, dreamy, sexy
Purple	Solemn, deep, mysterious, noble, arrogant, glamorous
Blue	Serenity, lost, peaceful, wisdom, hope, reason, transcendence, refreshing, eternal
Green	Hope, nature, balance, environmental protection, youth, growth, freshness
Light yellow	Quiet, serene, light-hearted
Yellow	Hope, joy, light, confidence, dignity, danger
Orange	Vitality, warmth, joy, kindness, joy, liveliness, leisure
White	Sublime, clean, parting, truth, indifference
Black	Simple, mysterious, composed, insidious, cold, evil, dead, noble

## Data Availability

The labeled data sets used to support the findings of this study are available from the corresponding author upon request.
